# Assessment of the Efficacy of Bone Marrow-Derived Mesenchymal Stem Cells against a Monoiodoacetate-Induced Osteoarthritis Model in Wistar Rats

**DOI:** 10.1155/2022/1900403

**Published:** 2022-08-16

**Authors:** Hadeer Mohamed Hamdalla, Rasha Rashad Ahmed, Sanaa Rida Galaly, Osama Mohamed Ahmed, Ibrahim A. Naguib, Badrah S. Alghamdi, Manal Abdul-Hamid

**Affiliations:** ^1^Cell Biology, Histology and Genetics Division, Department of Zoology, Faculty of Science, Beni-Suef University, P.O. Box 62521, Beni Suef, Egypt; ^2^Physiology Division, Zoology Department, Faculty of Science, Beni-Suef University, P.O. Box 62521, Beni Suef, Egypt; ^3^Department of Pharmaceutical Chemistry, College of Pharmacy, Taif University, P.O. Box 11099, Taif 21944, Saudi Arabia; ^4^Department of Physiology, Neuroscience Unit, Faculty of Medicine, King Abdulaziz University, Jeddah 22252, Saudi Arabia; ^5^Pre-Clinical Research Unit, King Fahd Medical Research Center, King Abdulaziz University, Jeddah, Saudi Arabia

## Abstract

Osteoarthritis (OA) of the knee is a debilitating condition that can severely limit an individual's mobility and quality of life. This study was designed to evaluate the efficacy of bone marrow-derived mesenchymal stem cell (BM-MSC) treatment in cartilage repair using a rat model of monoiodoacetate- (MIA-) induced knee OA. OA was induced in the knee joint of rats by an intracapsular injection of MIA (2 mg/50 *μ*L) on day zero. The rats were divided into three groups (*n* = 6): a normal control group, an osteoarthritic control group, and an osteoarthritic group receiving a single intra-articular injection of BM-MSCs (5 × 10^6^ cells/rat). The knee diameter was recorded once per week. By the end of the performed experiment, X-ray imaging and enzyme-linked immunosorbent assay analysis of serum inflammatory cytokines interleukin-1beta (IL-*β*), IL-6, and tumor necrosis factor-*α* (TNF-*α*) and anti-inflammatory cytokines interleukin-10 and transforming growth factor-beta (TGF-*β*) were carried out. In addition, RT-PCR was used to measure nuclear factor-kappa B (NF-*κ*B), inducible nitric oxide synthase (iNOS), and type II collagen mRNA levels and Western blot analysis was used to determine caspase-3 protein levels in all treated groups. Finally, hematoxylin/and eosin stains were used for histopathological investigation. Administration of BM-MSCs significantly downregulated knee joint swelling and MIA-induced (IL-1*β*, IL-6, and TNF-*α*) and upregulated IL-10 and TGF-*β* as well. Moreover, BM-MSC-treated osteoarthritic rats exhibited decreased expression of NF-*κ*B, iNOS, and apoptotic mediator (caspase-3) and increased expression of type II collagen when compared to rats treated with MIA alone. The hematoxylin/eosin-stained sections revealed that BM-MSC administration ameliorated the knee joint alterations in MIA-injected rats. BM-MSCs could be an effective treatment for inflamed knee joints in the MIA-treated rat model of osteoarthritis, and the effect may be mediated via its anti-inflammatory and antioxidant potential.

## 1. Introduction

Knee osteoarthritis (OA) is a disorder that influences the musculoskeletal system in youth and the elderly [1]. It is a degenerative joint disease, which is marked by pain, erosion of articular cartilage, osteophytes, subchondral sclerosis, and a variety of biochemical and morphologic changes that occur in the synovial membrane and joint capsule [2]. The rapid increase of OA is expected to significantly impact health care and public health systems in the future. With an aging population, the physical and economic burden of OA is tremendous as it is considered one of the main reasons for disability among the elderly [1, 3].

The pathogenesis of diseases of joints such as OA is associated with progressive degeneration of articular cartilage, bone remodeling, and locally produced cytokines, chemokines, and other inflammatory mediators by synovium and chondrocytes. Up to date, it is not clear to determine strictly the exact cause of OA specifically and OA progression risk depends on a wide range of factors. The dysbacteriosis of the gut microbiota can be claimed to be a predisposing factor for OA pathogenesis since it leads to obesity, insulin resistance, and systemic inflammation [4]. However, most attempts at treatment have only been effective at reducing the disease symptoms (pain relief) [5].

Despite extensive work, there is currently no treatment that can cure or effectively slow the progression of OA [6]. Because the efficacy of new therapeutics is initially tested in animal models of OA [7], it is important to develop animal models that accurately depict joint pathogenesis and treatment response and provide useful biomechanical, radiological, and microscopic assessments of OA-affected tissues [8]. The monoiodoacetate- (MIA-) induced model of OA, as opposed to surgical models, is an ideal experimental model that is easy to generate, and it induces OA alterations similar to those observed in humans [9]. It exhibits increased inflammatory cytokines and decreased anti-inflammatory cytokines, thereby mimicking the inflammation process [10].

Current studies have focused on mesenchymal stem cell (MSC) therapies as they promote the protection, regeneration, and restoration of degenerated and injured joints resulting from arthritis [11–13]. Although the precise mechanism underlying the effectiveness of stem cell-based injectable treatments is not yet completely known [14], the capability of MSCs to migrate and engraft onto multiple musculoskeletal tissues and undergo differentiation into functional chondrocytes [15, 16], regenerate meniscus [17], and produce therapeutic growth factors and cytokines [6, 18] has drawn significant interest as a way to facilitate the repair of damaged tissues and halt disease progression. Consequently, the main objective of the presented work is to evaluate the ability of bone marrow-derived mesenchymal stem cells (BM-MSCs) to repair deterioration in the articular cartilage in MIA-induced osteoarthritis in a rat model utilizing radiographic, biochemical, and real-time polymerase chain reaction (RT-PCR), Western blot, and histological analyses.

## 2. Materials and Methods

The experiments were performed using eighteen adult male Wistar rats (weighing 130–150 g). They were brought from the animal house of Al-Nahda University, Beni Suef, Egypt, maintained under conditions of controlled humidity, fed with commercial rat pellets and water ad libitum, and their weight was measured weekly. All procedures followed the guidelines of the “experimental animal ethics committee” of the faculty of science, Beni-Suef University, Egypt, for the use and care of animals, and the ethical approval number is BSU/FS/2018/15.

### 2.1. Induction of Osteoarthritis (OA)

The osteoarthritis model was constructed on day zero (Figure 1). The left knees of twelve rats were sprayed with 70% alcohol and then intra-articularly injected with 50 *μ*L of sterile saline (0.9%) containing monosodium iodoacetate (MIA) (2 mg/50 *μ*L) using a 21-gauge needle as previously described by Maresca et al. [19].

### 2.2. Isolation and Culture of Bone Marrow Mesenchymal Stem Cells

The protocol for the isolation and culture of BM-MSCs was done according to the procedure of Ahmed et al. [11] and Chaudhary and Rath [20]. BM-MSCs were flushed out of the humerus, femurs, and tibiae of the rats and centrifuged at 3000 RPM for 5 min at room temperature. They were cultured in culture flasks containing Dulbecco's modified Eagle's medium (DMEM) (Life Science Group Ltd., UK) supplemented with 10% fetal bovine serum (Lonza Verviers Sprl, Belgium), 0.36% sodium hydrogen carbonate, and 1% penicillin/streptomycin (Life Science Group Ltd., UK) and kept at 37°C in a 5% CO_2_ incubator. On the third day, the culture medium was changed. After 7–10 days, the cells were collected using trypsin (Greiner Bio-One, Germany).

### 2.3. Viability Assessment

For cell counting and viability assessment, the collected cells were washed and resuspended in DMEM. Then, 10 *μ*L of 0.4% trypan blue was added to 10 *μ*L of the cells and the mixture was counted on a hemocytometer. The BM-MSCs dispersed in DMEM with viability higher than 95% were immediately injected into the knee joint of osteoarthritic rats at a dose of 5 × 10^6^ cells/rat.

### 2.4. Animal Grouping and Experimental Design

Eighteen adult male Wistar rats were randomly selected and categorized into the following three groups (*n* = 6) (Figure 1):

#### 2.4.1. G1 (Normal Control Group)

The rats within the control group received an intracapsular injection of saline (50 *μ*L) and DMEM (50 *μ*L) into the left knee joint at 0 and 14 days.

#### 2.4.2. G2 (MIA-Induced OA Group)

The rats within this group were administered a single intra-articular injection of 50 *μ*L saline containing 2 mg MIA [19] and 50 *μ*L of DMEM into the left knee joint at 0 and 14 days.

#### 2.4.3. G3 (MIA + BM-MSC Group)

On the 14^th^-day post-MIA injection, the rats were treated using a single intra-articular injection (50 *μ*L) of BM-MSCs at a dose of 5 × 10^6^ cells/joint [21].

#### 2.4.4. Knee Measurement

The differences in the measurements of the anterior-posterior diameters of the affected and unaffected knee joints were measured using a manual caliper [22]. The measurements were recorded on day zero and every week post-MIA injection until the end of the experiment. Then, the mean variance in the volume of injected knee edema (swelling) relative to the noninjected knee was obtained.

#### 2.4.5. Radiographic Assessment (X-Ray)

On day 27 post-OA induction and day 14 post-BM-MSC treatment, the knee joints of haphazardly taken rats under anesthesia were X-rayed (anterior-posterior position) using an X-ray apparatus (Shimadzu Corporation, Japan) to observe impairment in joint space, bone morphology, and response to BM-MSC treatment.

#### 2.4.6. Blood and Tissue Samples

After 28 days, animals were anesthetized with diethyl ether inhalation and blood samples were collected from the jugular vein. Obtained blood was left to coagulate at ambient temperature for 30 min, followed by centrifugation at 3000 rpm for 15 min. Obtained serum was quickly removed and kept at −20°C until being used for the analysis of various biochemical parameters. Three knee samples from each group were fixed in 10% buffered formalin for histopathological evaluation, whereas the others were kept at −20°C until being utilized for RT-PCR and Western blot analysis.

#### 2.4.7. Enzyme-Linked Immunosorbent Assay Analysis

The amounts of serum tumor necrosis factor-*α* (TNF-*α*), interleukin-1 beta (IL-1*β*), IL-6, IL10, and transforming growth factor-beta (TGF-*β*) of all groups were defined using specific enzyme-linked immunosorbent assay kits supplied by MyBioSource (USA) according to the manufacturer's instructions.

#### 2.4.8. Antioxidant Defense System and Oxidative Stress Analysis

The glutathione (GSH) content, lipid peroxidation, and superoxide dismutase (SOD) activity were measured in serum as part of the antioxidant defense system. Later on, lipid peroxidation was determined following the method of Preuss et al. [23] based on the determination of malondialdehyde (MDA), which is an end product of lipid peroxidation reacting with thiobarbituric acid (TBA) to yield a pink-colored TBA-reactive substance, which assesses the amount of lipid peroxidation. SOD activity was determined following the Nishikimi et al. [24] procedure. This assay relies on the ability of the enzyme to inhibit the phenazine methosulphate-mediated reduction of nitro blue tetrazolium dye. GSH levels were measured following the method of Beutler et al. [25]. It is the reduction of 5, 5′-dithiobis-2-nitrobenzoic acid (DTNB) by the thiol group (SH) which is present in GSH to form 5-thio-2-nitrobenzoic acid, where the latter can be assayed colorimetrically.

#### 2.4.9. Real Time-PCR (RT-PCR) Analysis

The QIAGEN tissue extraction kit (QIAGEN, USA) was used for total RNA isolation. Then, 0.5–2 *μ*g of total RNA was used for cDNA synthesis using a kit from Fermentas (USA). An Applied Biosystem instrument with software version 3.1 (StepOne™, USA) was for real-time qPCR amplification and analysis. The qPCR assay was done with primer sets optimized for the annealing temperature. The sequences of the primers are presented in Table 1.

#### 2.4.10. Western Blot Analysis

Western blot (WB) analysis was implemented to assess the amount of protein of NF-*κ*B p50, NF-*κ*B p65, caspase-3, and cleaved caspase-3 in the knee samples. Briefly, the proteins were extracted from the left knee joints (*n* = 3) using ice-cold radioimmunoprecipitation assay buffer (RIPA buffer) supplemented with protease and phosphate inhibitors (Bio Basic Inc., Canada). Equivalent amounts of protein (30 *μ*g) were isolated on 10% sodium dodecyl sulfate-polyacrylamide gels (SDS-PAGE). Furthermore, proteins were transferred to polyvinylidene fluoride (PVDF) membranes and blocked with 5% skim milk in TBS containing Tween 20 overnight. The membranes were incubated at 4°C with primary antibodies against NF-*κ*B p50, NF-*κ*B p65, caspase-3, and cleaved caspase-3. Following washing with TBST, membranes were incubated with the corresponding secondary antibodies and developed using an enhanced chemiluminescence kit (BioRad, USA). Finally, the developed blots were scanned and band intensity was measured using ImageJ software (NIH, USA).

#### 2.4.11. Histopathology of the Knee Joint

After dissection, 3 knee joint samples from each group were rapidly excised and trimmed for histopathological examination. They were fixed in 10% buffered formalin for 24 h and decalcified in 10% formic acid solution, dehydrated, and embedded in paraffin wax. After cutting into 5 *μ*m sections, the slides were stained with hematoxylin and eosin stain for examination by light microscopy. The histopathology of OA is graded using the modified Mankin grading system [26, 27] as follows: the cartilage structure was scored from 0 to 4 (Table 2), where 0 is normal, 1 is surface irregularities, 2 is complete disorganization, 3 is clefts into the noncalcified cartilage layer, and 4 is clefts into the calcified cartilage layer. Furthermore, cellular abnormalities were scored on a scale of 0 to 3, where 0 is normal, 1 is hypercellularity, including small superficial clusters, 2 is clusters, and 3 is hypocellularity. Finally, tidemark was graded on a scale of 0 to 1, where 0 is intact and 1 is damaged.

#### 2.4.12. Statistical Analysis

All the data were presented as the mean ± SEM, where *P* < 0.05 was deemed statistically significant. All values were analyzed by IBM-SPSS software (version 25.0) using one-way ANOVA followed by post hoc Dunnett's *t*-test at different variance levels.

## 3. Results

### 3.1. Effect of BM-MSCs on Knee Diameter Measurements

The MIA-treated group showed an increase in knee diameter during the first two weeks post-MIA injection compared with the values on day zero before MIA injection. However, MIA rats treated with BM-MSCs on day 14 exhibited a reduction in the knee measurement throughout the third and fourth weeks of the experiment compared to the MIA-treated group (Figure 2).

### 3.2. Effect of BM-MSCs on Radiographic Changes

At the end of the treatment period, the anterior and posterior views of the left knee joints from all groups were X-rayed. Compared with those of the normal rats (Figure 3(a)), the knees of the MIA-treated group showed OA alterations, such as cartilage degradation as evidenced by the existence of bone erosions, a narrow joint space, and minute marginal osteophytes (Figure 3(b)). In contrast, the BM-MSC-treated knees exhibited a significant restoration of normal joint morphology, marked by the recovery of joint space narrowing and disappearance of osteophytosis osteophytotic (Figure 3(c)).

### 3.3. ELIZA Evaluation

- Effect of BM-MSCs on the serum proinflammatory cytokines TNF-*α*, IL-1*β*, and IL-6

A remarkable increase (*P* < 0.05) in the serum levels of TNF-*α*, interleukin-1 beta (IL-1*β*), and IL-6 (Table 3) was observed in the MIA-treated group in comparison with the normal control group. On the contrary, the MIA + BM-MSC group had a significant decrease (*P* < 0.05) in the serum levels of TNF-*α*, IL-1*β*, and IL-6 in comparison with the MIA group.

(b) Effect of BM-MSCs on serum IL-10

The serum levels of IL-10 (Table 3) were markedly reduced in the osteoarthritic control group in comparison with the normal control group (*P* < 0.05), whereas the serum levels of IL-10 were remarkably increased (*P* < 0.05) in the BM-MSC-treated group compared with the MIA group.

(c) Effect of BM-MSCs on serum transforming growth factor-beta (TGF-*β*)

MIA administration had significantly increased the serum levels of TGF-*β* (Table 3) compared with the normal control rats. In contrast, the MIA + BM-MSC-treated group showed a reduction (*P* < 0.05) in the levels of TGF-*β* compared with the MIA-treated group and an increase relative to the normal rats.

### 3.4. Effect of BM-MSCs on Serum Levels of Malondialdehyde (MDA), Superoxide Dismutase (SOD), and Glutathione (GSH)

MIA-induced osteoarthritic rats had significantly (*P* < 0.05) increased MDA levels and decreased the activity of SOD and the concentration of GSH (Table 4). On the other hand, BM-MSC-treated rats exhibited a significant decrease in MDA levels accompanied by an elevation in the activity of SOD and the content of GSH.

### 3.5. Effect of BM-MSCs on mRNA Expression Levels of Nuclear Factor-Kappa B (NF-*κ*B), Inducible Nitric Oxide Synthase (iNOS), and Type II Collagen

The role of BM-MSC administration in osteoarthritic rats on the expression of nuclear factor-kappa B (NF-*κ*B), inducible nitric oxide synthase (iNOS), and type II collagen was determined by qRT-PCR (Figures 4–6), respectively. MIA administration markedly increased the expression of NF-*κ*B and iNOS in comparison with the normal control group. On the contrary, the BM-MSC treatment of osteoarthritic rats significantly inhibited the expression levels of NF-*κ*B and iNOS compared with the group treated with MIA only. On the other hand, BM-MSCs enhanced the expression of collagen type II mRNA compared to that of the osteoarthritic control group, which exhibited low expression of collagen type II.

### 3.6. Effect of BM-MSCs on the Protein Expression Levels of NF-*κ*B p50 and NF-*κ*B p65

Western blot analysis demonstrated the MIA-induced increase in the protein expression levels of NF-*κ*B p50 and NF-*κ*B p65 (Figure 7) in the knee joints of osteoarthritic rats relative to the normal knee joints, whilst MIA + BM-MSC-treated knee joints showed significant reduction in protein expression levels of NF-*κ*B p50 and NF-*κ*B p65 compared with the MIA-treated knee joints without any treatment.

### 3.7. Effect of BM-MSCs on the Protein Expression Levels of Caspase-3 and Cleaved Caspase-3

Western blot analysis revealed that the protein levels of cleaved caspase-3 and caspase-3 (Figure 8) were markedly enhanced in the knee joints of osteoarthritic rats in comparison with the normal rats. Furthermore, the upregulated protein levels of caspase-3 and cleaved caspase-3 were significantly attenuated in knee joints of osteoarthritic rats treated with BM-MSCs compared with the osteoarthritic control group.

### 3.8. Effect of BM-MSCs on Histopathological Changes

Hematoxylin and eosin sagittal stained sections of the normal knee revealed a normal histological composition of the joint capsule, articular cartilage, and subchondral bone as well as intact tidemarks (Figure 9(a)). In contrast, the stained sections of the osteoarthritic rats (MIA group) showed significant histopathological alterations in the cartilage including a reduction in thickness, clefting, uneven articular surface, and degenerated chondrocytes accompanied by apoptosis (Figure 9(b)). Osteoarthritic rats (Figure 9(b)) also displayed bone destruction in the discontinuous thin cancellous bone trabeculae with blind ends and widening of the bone marrow space, which contained fewer hematopoietic cells as well as invisible tidemarks. Moreover, matrix changes included a severe loss, degeneration, and heterogeneous distribution of chondrocytes in the growth plate (Figure 9(c)). However, osteoarthritic rats treated with BM-MSCs exhibited no histopathological bone lesions. In contrast, osteoarthritic rats treated with BM-MSCs showed profound protection against OA-related articular cartilage defects and indicated no histopathological lesions in cartilage or bone compared with osteoarthritic knee joints (Figures 9(d) and 9(e)). Likewise, the total score of the modified Mankin system (Table 5) was significantly lower in the BM-MSC osteoarthritic-treated group (*P* < 0.05) in comparison with the osteoarthritic control group which confirms the protective properties of stem cell treatment against further destruction of the cartilage in OA knee joints.

## 4. Discussion

OA was considered for a long time as a noninflammatory wear and tear condition involving cartilage degeneration. However, it has become clear that it is a whole-joint disease in which catabolic processes cause cartilage degradation and inflammation, which plays a key role in the pathogenesis and development of OA [28].

Considering the limited reparability of cartilage [16, 29] and that no cure is currently available for OA [30], MSCs are regarded as an auspicious candidate for knee OA treatment because of their chondroprotective effects, chondrogenic potential, and paracrine effects [31–33], as well as their ability to enhance the production of various extracellular matrix (ECM) components [34, 35].

In the present study, we shed light on the possible underlying mechanisms of action of a single intra-articular injection of BM-MSCs as therapy for cartilage damage in an MIA-induced OA rat model (Figure 10).

Joint swelling is frequent in various kinds of arthritis and is driven by edema, which occurs as a result of leakage of fluid from endothelial cells of the blood vessels into the inflamed synovium [36]. The intrainjection of BM-MSCs resulted in a substantial reduction in the increased values of the left knee diameter post-MIA administration. Similarly, a study by Kehoe et al. [37] revealed that treatment with BM-MSCs reduced knee swelling, which was ascribed to alterations in permeability of synovial endothelial cells to soluble substances produced by the MSCs.

Our radiographic findings in harmony with de Morais et al. [8] and Jaleel et al. [38] illustrated that MIA-induced chondral injury along with inflammation resulted in osteophytosis, bone sclerosis, and a reduction in joint space, analogous to human osteoarthritis. Moreover, radiography images revealed that two weeks of treatment with BM-MSCs attenuated the effect of MIA and resulted in a direct regenerative effect on knee joint cartilage.

Because damaged cartilage is subjected to a progressive inflammatory environment [39], several inflammatory signaling pathways, including the nuclear factor-kappa B (NF-*κ*B), have been implicated in the control of OA [40].

The classical-canonical pathway of NF-*κ*B is stimulated in chondrocytes and synoviocytes of articular joints by mechanical stress or cytokines (IL-1*β* and TNF-*α*) (Figure 10). It is started with the activation of IB kinase (IKK), resulting in phosphorylation and degradation of I*κ*B*α* by the proteasome, and then, NF-*κ*B p65 as well as NF-*κ*B p50 protein is released and translocated from the cytoplasm to the nucleus [41].

Activated chondrocytes and synoviocytes subsequently produce a plethora of inflammation-related factors, including matrix metalloproteinase proteins, inducible nitric oxide synthase (iNOS), IL-1*β*, IL-6, and TNF-*α*, and these cytokines further activate the signaling cascade [42].

Our results indicated that BM-MSCs significantly suppressed NF-*κ*B p50, NF-*κ*B p65, TNF-*α*, IL-1*β*, and IL-6 in osteoarthritic rats (Figure 10). These findings are consistent with Mancuso et al. [43] and Wang et al. [44]. A study by Wang et al. [45] hypothesized that MSC administration displayed anti-inflammatory effects via lessening excess TNF-*α* (an activator of NF-*κ*B) and blocking the phosphorylation of the NF-*κ*B p65 subunit in spinal cord injury.

Moreover, BM-MSC treatment significantly elevated the serum levels of IL-10 which is considered an anti-inflammatory cytokine that possesses chondroprotective characteristics [46]. Moreover, it can induce the proliferation of chondrocytes [47] and ameliorate the severity of arthritis and cartilage degeneration [48]. The immunomodulatory capacity of activated MSCs alters inflammatory cytokine levels during OA and can affect IL-10 expression, which results in tissue survival [49]. Previous studies proposed that prostaglandin E2 (PGE2) released by MSCs can increase the secretion of IL-10 by engaging the E-type prostanoid receptors, EP2 and EP4 receptors, on M2 macrophages which eventually repair the damage of the cartilage [44, 50].

In our study, BM-MSC injection also markedly decreased inducible nitric oxide synthase expression in the osteoarthritic knee joints. Hamilton et al. [51] stated that intra-articular injection of MSC could downregulate the iNOS level in macrophages and eventually reduces the generation of M1 macrophages.

The expression of proinflammatory and damaging mediators of OA, such as the iNOS gene, has also been linked to NF-*κ*B signaling [52, 53]. iNOS is considered an enzyme responsible for the generation of nitric oxide (NO). Excessive production of NO by iNOS appears to be involved in OA pathogenesis through modulating ECM homeostasis and cytokine expression, which results in oxidative damage and chondrocyte apoptosis [54].

The immunosuppressive nature of MSCs may also explain the outcomes of iNOS levels in our study. Under inflammatory conditions, interferon *γ* (IFN*γ*), in combination with one of three additional proinflammatory cytokines, TNF-*α*, IL-1, or IL-1*β*, induces the immune activity of MSCs. In response to this cytokine combination, MSCs express multiple chemokines and iNOS, which directly prevent the proliferation and function of T cells [55].

Even though transforming growth factor-beta (TGF-*β*) signaling has a principal role in cartilage development and in maintaining articular chondrocyte homeostasis in synovial joints, in the present study, TGF-*β* is potentially involved in joint degeneration. Similarly, a study by Dranitsina et al. [56] revealed that MIA-OA causes an increase in the expression of Tgfb1 genes in rat cartilage cells. Our results, in contrast to Halfaya et al. [57], indicated a significant rise in the level of transforming growth factor *β* (TGF-*β*) in OA joints compared with that of the control group [46]. Van der Kraan [28] postulated that an elevation of the TGF-*β* level could activate inflammation that may be involved in OA pathogenesis by altering cellular differentiation and causing joint deterioration. Additionally, studies have reported that TGF-*β* signaling mediated by Smad2/3 may be involved in OA progression by inducing the recruitment of MSCs and osteoprogenitors to the subchondral bone, ending with aberrant bone remodeling that initiates and worsens osteoarthritis. Nevertheless, the activation and catabolic role of TGF-*β* in OA requires further investigation.

However, TGF-*β* levels after BM-MSC treatment were still higher compared with those of the normal control group. Studies have reported that MSCs could inhibit T-cell proliferation and promote apoptosis in T cells, ending with fragments that trigger phagocytes to release TGF-*β* [6, 58].

Apoptosis also plays a key role in OA pathophysiology. MIA has been shown to have necrotic and proapoptotic effects on rat chondrocytes in vitro, whilst TNF-*α* activates the tumor necrosis factor receptor (TNFR) or death receptors which eventually triggers the extrinsic pathway of apoptosis (Figure 10).

Korotkyi et al. [59] demonstrated that MIA-OA induced free radical reactions that caused the accumulation of superoxide anion radicals, hydrogen peroxide, and NO and thiobarbituric acid-reactive compounds that are intermediate products of lipid peroxidation. Elevated oxidative stress and ROS levels triggered by MIA led to the activation of the intrinsic pathway through the depolarization of membrane potential, the promotion of the discharge of cytochrome c, and the activation of caspase-3 [10, 60, 61]. Caspase-3 contributes to the overall apoptotic process by cleaving various cellular substrates [62]. Korotkyi et al. [59] also mentioned that MIA-induced OA led to a decrease in superoxide dismutase (SOD) activity of glutathione (GSH) which represents the first line of antioxidants that catalytically scavenge the free radicals [13].

Overall, MIA-OA condition results in an imbalance between the intensity of the formation of free radicals and their neutralization by the antioxidant defense system. Therefore, inhibiting ROS and caspase-3 expression in OA could potentially inhibit apoptosis.

In this context, we tested the effect of BM-MSC injection on the increase of the lipid peroxidation product (MDA) and the decrease of SOD and GSH levels in MIA-induced OA in the knee joints of the rat. Our data showed that the antioxidant system was boosted and that the increased level of caspase-3 and MDA in OA knee joints was ameliorated following intra-articular MSC treatment.

MSCs release an array of paracrine molecules, known as secretome, consisting of a variety of proteins with diverse biological functions, including immune regulation, antiapoptotic effects, and antioxidative effects. Antioxidant effects exhibited by MSCs and their secretome are attributed to their ability to scavenge free radicals, upregulate the antioxidant defense system, and alter cellular bioenergetics [63]. MSC immunosuppressive capabilities can also prevent the production of ROS and lower oxidative stress. Most recently, BM-MSCs decreased oxidative stress and enhanced antioxidant activity in severe acute pancreatitis in rats by inducing the nuclear translocation of nuclear factor erythroid 2-related factor 2, an emerging regulator of cellular resistance to oxidants, via the PI3K/AKT signaling pathway [64]. Meanwhile, He et al. [65] proposed that the paracrine effect of MSC mitigated ischemia-induced apoptosis by increasing the Bcl-2-to-Bax ratio and inhibiting the activation of caspase-3.

Oxidative stress and ROS have also been linked to OA pathophysiology by inhibiting new cartilage extracellular material (ECM) synthesis, leading to a loss of integrity of the cartilage [66]. The degradation and low accumulation of type II collagen, a predominant component of ECM that interacts with proteoglycans, supplying the cartilage with the elasticity and capacity for deformation, have been implicated in OA condition [67]. Besides, the newly produced molecules to compensate for the loss are often damaged which inhibits cartilage repair [68].

Lepetsos and Papavassiliou [54] suggested that ROS restrains mitochondrial oxidative phosphorylation and ATP formation in cultured chondrocytes, which eventually decreases the synthesis of collagen and proteoglycans and results in cartilage degradation.

On the other hand, MSCs have also been shown to promote chondrogenesis by replenishing the ECM of articular cartilage [35]. Intra-articular BM-MSC administration diminished the loss of collagen type II in OA knee joints. Ahmed et al. [13] have suggested that BM-MSCs could promote the antioxidant defense system at the expense of the oxidative stress in tissues, hence, inhibiting the subsequent inflammatory process (Figure 10).

Histopathological evaluation was the major endpoint examined in the current study. Four weeks post-MIA administration, the osteoarthritic control displayed multiple histopathological changes in the knee joint including severe damage to the cartilage structure which was manifested by a loss of integrity, clefts, degeneration of the surface layer, matrix changes, dispersed and pyknotic chondrocytes, and hypocellularity resulting from the loss and degeneration of chondrocytes [69, 70]. In the present study, a single intra-articular injection of BM-MSCs significantly lessened the inflammation and provided adequate protection against MIA-induced histopathological alterations, which were demonstrated by the preserved structure of articular cartilage, ECM, and the underlying subchondral bone [21, 71], However, the impact of a single injection of BM-MSC on cartilage regeneration and proliferation should be further studied. These results are also supported by the overall Mankin score as the rats, which received an intra-articular injection of BM-MSC showing a remarkable amelioration of the articular cartilage structure represented by a lower Mankin score compared with the osteoarthritic rats without treatment.

Considering the biochemical, molecular, and histopathological outcomes, our results suggest that BM-MSC treatment regulates and reduces OA-induced inflammation, postpones cartilage degradation, and promotes cartilage regeneration through paracrine activity [72].

Although this study has reached its aims, there were some potential limitations that the relevant mechanism underlying the effects of BM-MSCs on OA has not yet been further confirmed because of an insufficient small sample size and a lack of ability in predicting the pathway and safety in clinical investigations. In future studies of OA and treatments with BM-MSCs, researchers should focus on in-depth investigations of the various molecular mechanisms underlying OA and screening and identifying specific signaling pathways.

## 5. Conclusion

It was concluded that intra-articular injections of BM-MSCs significantly enhanced the radiological, biochemical, molecular, and histopathological outcomes of rats suffering from knee OA induced by MIA over a two-week period. However, cartilage regeneration probably takes a long time to develop. Therefore, to determine the long-term efficacy of BM-MSCs on the progress of knee OA, long-term studies should be carried out.

## Figures and Tables

**Figure 1:** Timeline of the experiment depicting OA induction on zero day, treatment on the 14^th^ day, and sacrifice of animals on the 28^th^ day.

**Figure 2:** Knee anterior-posterior diameter measurements in normal control, MIA, and MIA + BMMSC groups. At each period, the means, which have different symbols (letters), are significantly different at *P* < 0.05.

**Figure 3:** Radiographic changes in the left knee joint (L). (a) The normal control group shows a healthy knee joint with a smooth articular cartilage surface and normal joint space (arrowhead). (b) The MIA-treated group demonstrates OA alternations such as a remarkable narrowing of the joint space (arrowhead), erosion, subchondral sclerosis (curved arrow), and osteophyte (black arrow). (c) The MIA + BMMSC-treated group shows nearly restored normal joint space (arrowhead) and cartilage surface.

**Figure 4:** Effect of BM-MSC treatment (5 × 10^6^ cells/rat) on the mRNA expression level of NF-*κ*B in MIA-induced animals. Means, which have different symbols, are significantly different at *P* < 0.05.

**Figure 5:** Effect of BM-MSC treatment (5 × 10^6^ cells/rat) on the mRNA expression level of iNOS in MIA-induced osteoarthritic animals. Means, which have different symbols, are significantly different at *P* < 0.05.

**Figure 6:** Effect of BM-MSC treatment (5 × 10^6^ cells/rat) on the mRNA expression level of type II collagen in MIA-induced osteoarthritic animals. Means, which have different symbols, are significantly different at *P* < 0.05.

**Figure 7:** Effect of BM-MSC treatment (5 × 10^6^ cells/rat) on the protein levels of NF-*κ*B p50 and NF-*κ*B p65 in MIA-induced animals. Means, which have different symbols, are significantly different at *P* < 0.05.

**Figure 8:** Effect of BM-MSC treatment (5 × 10^6^ cells/rat) on the protein levels of cleaved caspase-3 and caspase-3 in MIA-induced animals. Means, which have different symbols, are significantly different at *P* < 0.05.

**Figure 9:** Photomicrographs of hematoxylin and eosin- (H&E-) stained sections of left knees joints of the following groups: (a) is a section from the control group which demonstrates the normal structure of articular cartilage, with a regular smooth intact surface and well-organized chondrocytes, which appeared in noncalcified (NCC) and calcified (CC) regions of cartilage with a clear intact tidemark (arrowhead) in between. The noncalcified region (NCC) of the articular cartilage is arranged in three zones: superficial (S), transitional (T), and radial (R) zones. It also shows intact subchondral bone (SC) with well-oriented bony trabeculae (arrow) (scale bar = 200 *μ*m). (b, c) Are sections from osteoarthritic rats (MIA-treated group). (b) Depicts clefting (curved arrows), surface erosion, degeneration of the surface layer with discontinuity of the matrix (star), discontinuous thin cancellous bone trabeculae having blind ends (arrows), decrease in thickness of articular cartilage, degenerated chondrocytes with pyknotic nuclei (arrowheads), and widening of bone marrow space (BM) containing less hemopoietic cells, invisible tidemark, and large, thickened area at the joint margin and disorganization of the articular cartilage with some cell clusters (thick arrow). (c) Shows the matrix change, loss, degeneration (∗), and heterogeneous distribution of chondrocytes in the growth plate. (d, e) Are sections from the treatment group (MIA + BMMSCs). (d) Displays intact synovial membrane (SV) and marked restoration of the normal structure of the articular cartilage intact surface and increase in its thickness and nearly normal bone marrow space (BM) compared to the MIA-treated group, organized fibrous connective tissue (thin arrows), clarification of tidemark (arrowhead), and cell layers with few shrunken chondrocytes, some empty lacunae (scale bar = 200 *μ*m). (e) Demonstrates neatly and normally oriented chondrocytes of the growth plate (scale bar = 200 *μ*m).

**Figure 10:** The therapeutic effect of BMMSCs on cartilage damage due to inflammation, extracellular matrix (ECM) degradation, and apoptosis in MIA-induced knee osteoarthritis.

**Table 1:** Primer sequences used for real-time PCR.

Target gene	Primer sequence
NF-*κ*B	Forward primer: 5′-CATTGAGGTGTATTTCACGG-3′ Reverse primer: 5′-GGCAAGTGGCCATTGTGTTC-3′
iNOS	Forward primer: 5′-GACCAGAAACTGTCTCACCTG-3′ Reverse primer: 5′-CGAACATCGAACGTCTCACA-3′
Type II collagen	Forward primer: 5′-GAGTGGAAGAGCGGAGACTACTG-3′ Reverse primer: 5′-CTCCATGTTGCAGAAGACTTTCA-3′
Beta-actin	Forward primer: 5′-TGTTTGAGACCTTCAACACC-3′ Reverse primer: 5′-CGCTCATTGCCGATAGTGAT-3′

**Table 2:** The modified Mankin score of microscopic observation of OA articular cartilage.

Category	Subcategory	Score
Structure	Normal	**0**
	Surface irregularities	**1**
	Complete disorganization	**2**
	Clefts to the noncalcified layer	**3**
	Clefts to calcified layer	**4**
Cells	Normal	**0**
	Hypercellularity	**1**
	Hypocellularity	**2**
	Pyknosis	**3**
Tidemarks	Intact	**0**
	Damaged	**1**

**Table 3:** Effect of BM-MSCs on serum levels of TNF-*α*, IL-6, IL-10, and TGF-*β* of MIA-induced OA.

Groups	Parameters				
	TNF-*α* (pg/mL)	IL-1*β* (pg/mL)	IL-6 (pg/mL)	IL-10 (pg/mL)	TGF-*β* (pg/mL)
Normal control	22.16 ± 1.62^a^	8.58 ± 3.14^a^	60.06 ± 2.97^a^	320.19 ± 2.33^c^	114.49 ± 0.52^a^
MIA	95.033 ± 0.71^c^	130.39 ± 3.95^c^	178.40 ± 5.86^c^	119.08 ± 3.71^a^	260.65 ± 6.62^c^
MIA + BM-MSCs	60.40 ± 2.05^b^	2.21 ± 4.95^b^	130.13 ± 8.50^b^	288.36 ± 1.54^b^	134.98 ± 3.88^b^

The number of samples in each group is six and the data are described as means ± SEM. For each parameter, means, which have different superscript symbols, are statistically significant, *P* < 0.05.

**Table 4:** Effect of BM-MSCs on serum levels of MDA, GSH, and the activity of SOD of MIA-induced OA.

Groups	Parameters		
	MDA (nmol/mL)	GSH (mg/dL)	SOD (U/mL)
Normal control	0.016 ± 0.004^a^	183.96 ± 16.26^c^	339.46 ± 13.49^c^
MIA	0.162 ± 0.037^c^	16.057 ± 2.9^a^	150.97 ± 11.08^a^
MIA + BM-MSCs	0.087 ± 0.006^b^	55.33 ± 5.98^b^	227.68 ± 8.33^b^

The number of samples in each group is six and the data are described as means ± SEM. For each parameter, means, which have different superscript symbols, are statistically significant, *P* < 0.05.

**Table 5:** Mankin scoring of the cartilage among experimental groups.

Groups	Parameters			
	Cartilage structure	Cellularity	Tidemarks	Overall Mankin score
Normal control	0 ± 0	0 ± 0^a^	0 ± 0^a^	0 ± 0^a^
MIA	4.0 ± 1.41^c^	1.26 ± 0.52^c^	1.0 ± 0.0^c^	11.17 ± 1.28^c^
MIA + BM-MSCs	2.50 ± 0.76^b^	0.55 ± 0.22^b^	0.33 ± 0.21^c^	4.17 ± 0.60^b^

The number of samples in each group is six and the data are described as means ± SEM. For each parameter, means, which have different superscript symbols, are statistically significant, *P* < 0.05.

## Data Availability

This published article includes all of the data generated or analyzed during this investigation.

## Abbreviations

BM-MSCs: Bone marrow-derived mesenchymal stem cells
DMEM: Dulbecco's modified Eagle's medium
DTNB: 5,5′-Dithiobis-2-nitrobenzoic acid
ECM: Extracellular matrix
MDA: Malondialdehyde
GSH: Reduced glutathione
IFN*γ*: Interferon *γ*
IL: Interleukin
iNOS: Inducible nitric oxide synthase
MIA: Monosodium iodoacetate
NF-*κ*B: Nuclear factor-kappa B
NO: Nitric oxide
OA: Osteoarthritis
PGE2: Prostaglandin E2
ROS: Reactive oxygen species
TBA: Thiobarbituric acid
TGF-*β*: Transforming growth factor-beta
TNFR: Tumor necrosis factor receptors
TNF-*α*: Tumor necrosis factor-*α*.
